# Human Action Recognition in Smart Cultural Tourism Based on Fusion Techniques of Virtual Reality and SOM Neural Network

**DOI:** 10.1155/2021/3495203

**Published:** 2021-12-03

**Authors:** Zaosheng Ma

**Affiliations:** School of Design and Art, Xijing University, Xi'an, Shannxi 710123, China

## Abstract

Smart cultural tourism is the development trend of the future tourism industry. Virtual reality is an important tool to realize smart tourism. The reality of virtual reality mainly comes from human-computer interaction, which is closely related to human action recognition technology. Therefore, the research takes human action recognition as the research direction, uses a self-organizing mapping network (SOM) neural network to extract the key frame of action video, combines it with multi-feature vector method to recognize human action, and compares the recognition rate and user satisfaction of different recognition methods. The results show that the recognition rate of multi-feature voting human action recognition algorithm based on SOM neural network is 93.68% on UT-Kinect action, 59.06% on MSRDailyActivity3D, and the overall action recognition time is only 3.59 s. Within six months, the total profit of human-computer interactive virtual reality tourism project with SOM neural network multi-eigenvector as the core algorithm reached 422,000 yuan, and 88% of users expressed satisfaction after use. It shows that the proposed method has a good recognition rate and can give users effective feedback in time. It is hoped that this research has a certain reference value in promoting the development of human motion recognition technology.

## 1. Introduction

Virtual reality technology lays the foundation for the development of smart cultural tourism, provides tourists with a new perspective, gives tourism users a sense of reality, and, at the same time, greatly reduces the resources consumed in building a variety of scenes in reality [1]. Smart cultural tourism combined with virtual reality technology broadens the inherent thinking of tourists, breaks the limitations of traditional cultural tourism, breaks through the space and time limitations of tourism in real life, and enables tourists to obtain more free interaction through three-dimensional information space [2]. Intelligent cultural tourism with the introduction of virtual reality technology, also known as virtual tourism, enables users to interact with the virtual system in a three-dimensional scene so as to obtain the reality of real tourism [3]. The higher the level of human-computer interaction performance, the higher the user's sense of reality. Human action behavior recognition is the key technology that directly determines the effect of human-computer interaction. Therefore, this paper focuses on human action behavior recognition technology, aiming to provide some help for the development of smart cultural tourism. A self-organizing mapping network (SOM) is a kind of low-dimensional discrete mapping generated by learning the data in the input space, which gradually optimizes the network with a competitive learning strategy. It has the self-organizing characteristics of the human brain and can identify the intrinsic related characteristics in a problem [4]. In view of this, this paper studies how to extract the key frames of human action video through the competitive learning characteristics of the SOM network and then uses the voting strategy of multi-feature classification results to carry out the final recognition of human action.

Scenic spots, landmarks, and cultural relics constitute the main link of tourism. In recent years, the deterioration of scenic spots and landmarks has become the main problem affecting the development of the tourism industry. Therefore, Liu proposed to carry out virtual secondary tourism in the innovative ways of virtual reality and mixed reality [5]. Virtual reality tourism provides consumers with the opportunity to experience virtual reality tourism destinations. Kim and Hall have built a hedonistic motivation model with consumer hedonistic behavior as the core and found that the degree of consumer perceived enjoyment directly affects the flow state of virtual reality tourism [6]. Willems et al. analyzed three kinds of virtual performance media, including photos, 360° video, and virtual reality and found that the score of virtual reality was the highest, and the human-computer interaction technology had the greatest impact on consumers' telepresence [7]. Bogicevic et al. discussed how to use virtual reality to provide a comprehensive tourism experience before a hotel stay. The research results show that virtual reality can better express the psychological image of experience and a stronger sense of existence [8]. Wei et al. collected the experience data of the virtual reality roller coaster and found that the sense of virtual reality has a positive impact on the overall theme park experience of tourists through regression analysis [9]. Based on the theory of extrinsic motivation and intrinsic motivation, Peng et al. distinguished consumers' perception of virtual reality devices and virtual reality content and find that the experience effect of virtual reality directly affects tourists' travel intention [10].

The world of human existence belongs to a multi-sensory world. Digital interaction is mainly based on audio-visual elements, Shen et al. believe that as a sensory support technology, virtual reality promotes the integration of sensory input and enhances multi-sensory digital experience [11]. Buhalis et al. proposed that in the future service experience, we should pay attention to supersensory experience, superpersonalized experience, and beyond automation experience [12]. Pradhan et al. made an overall investigation and analysis on the development history of human-computer interaction technology in virtual reality and summarized the areas still to be discussed [13]. Shi et al. proposed a computer holographic model based on deep learning, which not only ensures the capability of continuous depth sense in the 3D scene but also promotes the further development of virtual reality and human-computer interaction [14]. Amabilino et al. proposed a new paradigm for deriving the energy function of high-dimensional molecular systems, generating data for low dimensional systems in virtual reality [15]. Jasrotia and Gangotia proposed the use of generalized regression neural network to generate the overall human motion so as to improve the accuracy of human motion recognition [16]. Gao et al. proposed a human motion recognition model based on the image domain pretraining model, which realized the distinction of small motion frame order [17]. Gurbuz and Amin believe that deep learning has great application value in target classification, so a human action recognition model based on deep learning is proposed to observe human activities, falls, and abnormal gait monitoring [18].

To sum up, in recent years, there are many researches on artificial neural networks, virtual reality, human-computer interaction, intelligent tourism, and so on, but the research on virtual reality tourism combined with SOM neural network fusion is insufficient [19]. Therefore, the experiment focuses on the correlation analysis of the SOM neural network, which is the key to smart cultural tourism and virtual reality.

The key SOM neural network research on smart cultural tourism and virtual reality emphasizes the combination of virtual reality with smart tourism, and the key frame extraction technology of key SOM neural networks can well realize the action target recognition in the landscape area. It is undeniable that the SOM network can reduce noise and redundant data in key frame extraction and greatly improve the recognition accuracy of group activities in the tourism landscape.

This research takes human motion recognition as the research direction, innovatively uses a self-organizing mapping network (SOM) neural network to extract the key frames of motion video, and combines it with multi-feature vector method to recognize human motion. The recognition rate and user satisfaction of different recognition methods are compared. Experimental results show that this method has a good recognition rate and can provide effective feedback to users in time. The multi-feature vector recognition method based on SOM neural network proposed in this paper can achieve a better recognition effect in action recognition and bring more real experiences to users.

## 2. Research on Motion Feature Extraction and Human Behavior Recognition Technology

### 2.1. Human Motion Feature Extraction

The key to realizing virtual reality tourism lies in human action recognition technology. Human action recognition is the process that the computer extracts the action feature vector according to the actual action data of the human body and understands the action [20]. Human action recognition mainly consists of the steps of detecting moving objects in image frames, extracting action features from image frames, and understanding action features.

As shown in Figure 1, Kinect belongs to depth sensor equipment, which is used to extract the human skeleton model in the research. Firstly, the motion trajectory of joint points is calculated; then the adjacent joint angle, central joint angle, and angular velocity of the central joint are calculated in turn; and finally, the human motion feature is extracted.

In Figure 2, the human joint points of the human skeleton are numbered *J*_*i*_ (*i* = 1, 2,…, 20); the joint points of the head are numbered *J*_1_; and the corresponding coordinates are (*x*_1_, *y*_1,_ and *z*_1_). In the human skeleton model, there are 20 joint points. After removing *J*_3_, *J*_4_, and the other two joint points that constitute the central vector, the remaining 18 joint points can construct 18 structure vectors.

(1) $$\begin{array}{c} \langle \overset{⟶}{a},\overset{⟶}{b}\rangle =\arccos\frac{\overset{⟶}{a}•\overset{⟶}{b}}{\left|\overset{⟶}{a}\right|\left|\overset{⟶}{b}\right|}. \end{array}$$

Equation (1) is the expression of the central joint angle of a joint point in motion, and $\overset{⟶}{a},\overset{⟶}{b}$ is the two vectors constituting the included angle $\langle \overset{⟶}{a},\overset{⟶}{b}\rangle$.

(2) $$\begin{array}{c} \Delta \alpha =\alpha_{2}-\alpha_{1}. \end{array}$$

Equation (2) is the expression of the angular velocity of the central joint, where *a*_1_ is the joint angle in the *t*_1_ frame, *a*_2_ is the joint angle in the *t*_2_ frame, and △*a* is the angle change from frame *t*_1_ to frame *t*_2_. When the video frame rate is *f*(fps), the time interval Δ*t* expression of joint angle change can be obtained by sampling once per frame, as shown in the following equation:

(3) $$\begin{array}{c} \Delta t=\frac{n}{f}. \end{array}$$

Combining (2) and (3), the angular velocity *v*=Δ*α*/Δ*t* can be obtained. By combining the angular velocity of the *j* frame, the angular velocity eigenvector *D*_*j*_ (*j* = 1, 2,…, *F*) of the frame can be obtained. *F* refers to the total number of frames, and then the central angular velocity eigenvector *D(D*_1_, *D*_2_,…, *D*_*F*_) can be obtained.

(4) $$\begin{array}{c} P_{j}=\left[p_{j,1},p_{j,2},\ldots ,p_{j,t},\ldots ,p_{j,F}\right]. \end{array}$$

In (4), the coordinate (*x*_*t*_, *y*_*t*_, and *z*_*t*_) corresponding to the related node *j* at frame *t* is represented by *P*_*j, t*_, *t* ∈ *[*1, 2,…, *F]*, *t* ∈ *[*1, 2,…, 20*]*.

(5) $$\begin{array}{c} P=\left[\begin{array}{c} P_{1}\\ \vdots \\ P_{j}\\ \vdots \\ P_{20} \end{array}\right]=\left[\begin{array}{ccccc} p_{1,1} & \cdots & p_{1,t} & \cdots & p_{1,F}\\ \vdots & \vdots & \vdots & \vdots & \vdots \\ p_{j,1} & \cdots & p_{j,t} & \cdots & p_{j,F}\\ \vdots & \vdots & \vdots & \vdots & \vdots \\ p_{20,1} & \cdots & p_{20,t} & \cdots & p_{20,F} \end{array}\right]. \end{array}$$

Equation (5) is the motion trajectory expression of an action (20 joint points). The motion trajectory matrix is represented by *P*; the motion trajectory of joint points is represented by *p*_*j*_; and *p*_1*, t*_ is the three-dimensional coordinates of the first joint point in frame *t*.

(6) $$\begin{array}{c} G_{j}=\left[g_{j,1},g_{j,2},\ldots ,g_{j,t},\ldots ,g_{j,F}\right]. \end{array}$$

Equation (6) is the change matrix of adjacent joint angle corresponding to joint point *j*; the change process is represented by *G*_*j*_; and the size of adjacent joint angle corresponding to node *j* in *t* frame is represented by, where *F* is the total number of frames. It can be seen from Figure 2 that *J*_1_, *J*_5_, *J*_9_, *J*_13_, and *J*_17_, and other joint points have no corresponding adjacent joint angles, while *J*_2_, *J*_4_ corresponds to multiple adjacent joint angles.

(7) $$\begin{array}{c} G=\left[\begin{array}{c} G_{1}\\ \vdots \\ G_{j}\\ \vdots \\ G_{18} \end{array}\right]=\left[\begin{array}{ccccc} g_{1,1} & \cdots & g_{1,t} & \cdots & g_{1,F}\\ \vdots & \vdots & \vdots & \vdots & \vdots \\ g_{j,1} & \cdots & g_{j,t} & \cdots & g_{j,F}\\ \vdots & \vdots & \vdots & \vdots & \vdots \\ g_{18,1} & \cdots & g_{18,t} & \cdots & g_{18,F} \end{array}\right]. \end{array}$$

Equation (7) is a matrix expression of human action. In a certain frame, the coordinates corresponding to joint point *J*_1_ are (*x*_1_, *y*_1_, and *z*_1_), joint point *J*_2_ are (*x*_2_, *y*_2_, and *z*_2_), and joint point *J*_3_ are (*x*_3_, *y*_3_, and *z*_3_).

(8) $$\begin{array}{c} \overset{⟶}{J_{2}J_{1}}=\left\{x_{1}-x_{2},y_{1}-y_{2},z_{1}-z_{2}\right\}, \end{array}$$

(9) $$\begin{array}{c} \overset{⟶}{J_{2}J_{3}}=\left\{x_{3}-x_{2},y_{3}-y_{2},z_{3}-z_{2}\right\}. \end{array}$$

Equations (8) and (9) are the vectors after subtracting the coordinates. In this case, the expression of adjacent joint angle composed of two vectors can be obtained.

(10) $$\begin{array}{c} \langle \overset{⟶}{J_{2}J_{1}},\overset{⟶}{J_{2}J_{3}}\rangle =\arccos\frac{\overset{⟶}{J_{2}J_{1}}\cdot \overset{⟶}{J_{2}J_{3}}}{\left|\overset{⟶}{J_{2}J_{1}}\right|\left|\overset{⟶}{J_{2}J_{3}}\right|}. \end{array}$$

The value of joint angle $\langle \overset{⟶}{J_{2}J_{1}},\overset{⟶}{J_{2}J_{3}}\rangle$ in (10) is 0°–180°. There are 18 structure vectors corresponding to 18 central joint angles.

(11) $$\begin{array}{c} C_{j}=\left[c_{j,1},c_{j,2},\ldots ,c_{j,t},\ldots ,c_{j,F}\right]. \end{array}$$

Equation (11) is the expression of the change process of the center angle; it is expressed as *C*_*j*_; and the size of the central joint angle corresponding to the structure vector composed of the related node *j* in *t* frame is represented by *t C*_*j,t*_, where *F* is the total number of frames.

(12) $$\begin{array}{c} C=\left[\begin{array}{c} C_{1}\\ \vdots \\ C_{j}\\ \vdots \\ C_{18} \end{array}\right]=\left[\begin{array}{ccccc} c_{1,1} & \cdots & c_{1,t} & \cdots & c_{1,F}\\ \vdots & \vdots & \vdots & \vdots & \vdots \\ c_{j,1} & \cdots & c_{j,t} & \cdots & c_{j,F}\\ \vdots & \vdots & \vdots & \vdots & \vdots \\ c_{18,1} & \cdots & c_{18,t} & \cdots & c_{18,F} \end{array}\right]. \end{array}$$

Equation (12) is the schematic matrix of the change process of the central angle with time, and the angular velocity of the central joint corresponding to the joint point *j* that changes with the number of frames is *D*_*j*_.

(13) $$\begin{array}{c} D_{j}=\left[d_{j,1},d_{j,2},\ldots ,d_{j,t},\ldots ,d_{j,F}\right]. \end{array}$$

In (13), the angular velocity of the central joint corresponding to *j* in frame *t* is expressed by *d*_*j,t*_, where *F* is the total number of frames.

(14) $$\begin{array}{c} D=\left[\begin{array}{c} D_{1}\\ \vdots \\ D_{j}\\ \vdots \\ D_{18} \end{array}\right]=\left[\begin{array}{ccccc} d_{1,1} & \cdots & d_{1,t} & \cdots & d_{1,F}\\ \vdots & \vdots & \vdots & \vdots & \vdots \\ c_{j,1} & \cdots & c_{j,t} & \cdots & d_{j,F}\\ \vdots & \vdots & \vdots & \vdots & \vdots \\ d_{18,1} & \cdots & d_{18,t} & \cdots & d_{18,F} \end{array}\right]. \end{array}$$

Equation (14) is the change matrix of angular velocity corresponding to the central angle. According to different motion states, the corresponding angular velocity of human skeleton joint angle, the size of adjacent angle, and the change of central joint angle are used to extract motion features in different video frames.

## 3. Human Action Recognition Based on Voting Strategy of Multi-Feature Classification Results Combined with SOM

The human action is inconsistent at different times, so the motion feature data extracted from different frames are redundant. At the same time, the noise generated in the process of motion will also lead to the decline of the accuracy of human action recognition [21]. Therefore, SOM neural network is proposed to extract key frames of moving video.

As shown in Figure 3, SOM neural network is composed of input and competition layers. The two layers are connected with each other [22]. The neurons in each input layer are competitively responded by the neurons in the competition layer, and only one of them succeeds in the end. In the process of continuous competition, the weights of neurons in the network competition layer are constantly adjusted, and the expected results are finally output. Input the matrix **X** composed of all the eigenvectors of an action; initialize the winning field *N*_*j∗*_(0), learning rate *η*_0_, and learning rate threshold *η*_min_; set the total number of iterations iter; randomly assign the weight *w*_*j*_=(*j*=1,2,…, *m*) to each neuron in the competition layer; and obtain the weight vector **W** by combining the weights.

$\hat{W}=\left({\hat{w}}_{1},{\hat{w}}_{2},\ldots ,{\hat{w}}_{m}\right)$ exists in different elements of normalization **W**. Normalize the input eigenvector *t*=1, *N*_*j∗*_(*t*)=*N*_*j∗*_(0), and *η*_*t*_=*η*_0_ to get **X**_*i*_(1 ≤ *i* ≤ *F*) and calculate the dot product between ${\hat{X}}_{i}$ and $\hat{W}=\left({\hat{w}}_{1},{\hat{w}}_{2},\ldots ,{\hat{w}}_{m}\right)$. When the dot product is maximum, the corresponding neuron *j* is the winning neuron.

(15) $$\begin{array}{c} {\text{Dis}}_{j}=\exp\left(\frac{-S^{2}{}_{j,I\left(x\right)}}{2\eta^{2}}\right). \end{array}$$

Equation (15) is the updated weight Dis_*j*_ of neuron *j*; the index of winning neuron is *I*(*x*); and the distance between neuron *j* and winning neuron *j* is *S*_*j*,*I*(*x*)_.

(16) $$\begin{array}{c} w_{ij}=w_{ij}+\eta \left(t\right)\cdot {\text{Dis}}_{j}\cdot \left(x_{i}-w_{ij}\right). \end{array}$$

Equation (16) is the updated formula of the weights of neurons in the field. The weights of neurons *j* in the competition layer corresponding to ${\hat{X}}_{i}$ data in the input layer are expressed by *w*_*ij*_. The learning rate is updated according to *η*(*t*+1)=*η*_0_ · exp(−*t*/*η*(*t*)) and the neighborhood *N*_*j∗*_(*t*+1)=*N*_*j∗*_(0) · exp(−*t*/*N*_*j∗*_(*t*)).

As shown in Figure 4, after inputting the action feature vector obtained from the action video frame sequence into the self-organizing mapping network (SOM), through competitive learning, the trained weights of neurons in the competitive layer can be obtained [23]. The Euclidean distance between the weights of different neurons in the competitive layer of the feature vector and SOM neural network is obtained [24–31]. According to the Euclidean distance, the feature vectors are classified into different neurons; the last neuron is traversed to find out the nearest feature vector of each non-control neuron as the key frame [32–39].

The single feature action recognition technology has low reusability and low scalability. Therefore, based on the key frames extracted from the action video by SOM, through voting strategy, combined with the complementarity of different features, this paper improves the accuracy of human action recognition, increases the real sense of virtual reality, and improves the degree of virtual tourism enjoyment of tourists [40].

As shown in Figure 5, firstly, the feature vector corresponding to the feature of category I is read to construct the kernel function. Support vector machine (SVM) is used for classification, and the credit degree of feature I to different types of actions is calculated after classification. When all the class features are read, vote on the credit degree of different actions according to the classification results corresponding to different features and find out the action with the most votes or the action with the most credit degree.

If the recognition action type is *A*, the feature has been used for *E* action recognition in the past, and the action category of the *j* experiment is made into a sequence *Tlb*[*j*]; the recognition result sequence is *Plb*[*j*]; there are 1 ≤ *i* ≤ *A*, 1 ≤ *j* ≤ *E*, and action *i*; the number of correct recognition times is *EQ*_*i*,*j*_; and the total number of recognition times of action *i* in the *j* experiment is *LE*_*i*,*j*_.

(17) $$\begin{array}{c} {\text{acc}}_{i,j}=\frac{\sum_{j=1}^{E}EQ_{i,j}}{\sum_{j=1}^{E}LE_{i,j}}. \end{array}$$

(17) shows that in the *j* experiment, when the action *i* is recognized by this feature, the accuracy of recognition is *acc*_*i*,*j*_, and there is acc_*i*,*j*_ ∈ [0,1].

(18) $$\begin{array}{c} {\text{acc}}_{i}=\frac{\sum_{j=1}^{E}{\text{acc}}_{i,j}}{E}. \end{array}$$

Equation (18) shows that the recognition rate of action *i* is acc_*i*_ in all experiments.

## 4. Application Effect of Smart Cultural Tourism Based on SOM Neural Network

### 4.1. Effect Analysis of Human Action Recognition

Self-organizing mapping (SOM) is an unsupervised learning neural network used to solve the traveling salesman problem (TSP). Two-dimensional position coordinates are the input of the neural network, and spatial position relationship is the model to be learned by a neural network. The outgoing layer is usually a two-dimensional neuron grid (this paper is a one-dimensional ring structure). The data input from the input layer represents the pattern of the real world. The training goal of SOM is to map the pattern of the input data to the output layer. In the training, the weight vector of the output layer neurons will be updated, and the output layer neurons gradually learn the pattern behind the input data in the training.

The system development environment is Intel Core i5-6500; the memory size is 8G DDR4; and the operating system is Windows 7, 64-bit system. The experimental simulation is carried out on MATLAB R2016a. On the UT-Kinect motion data set, this paper uses semiconductor sensors to verify the recognition accuracy of the proposed multi-feature voting human motion recognition algorithm based on the SOM neural network. Firstly, the model is trained, as shown in Figure 6.

As can be seen from Figure 6, the system loss value of the SOM network decreases with the increase of the number of iterations, which shows that the error rate of the model decreases with the increase of the number of iterations. And it is not difficult to see that the increase in the number of iterations leads to the continuous improvement of the accuracy of the network model. Secondly, the action is recognized by a single feature, and then the action is recognized by the algorithm. Finally, the recognition rate of the two methods is compared.

As shown in Figure 7, through the research of the proposed multi-feature voting human action recognition algorithm based on SOM neural network, the average accuracy rate of action recognition in UT-Kinect action data set is 93.68%, which is 1.04% higher than that based on joint point coordinates. The accuracy rate of human action recognition based on a center angle is 82.64%. The accuracy rate of human action recognition based on the center angular velocity is 67.39%. The accuracy of human action recognition based on the single feature of adjacency angle is 83.82%; The results show that the recognition accuracy of the proposed method is higher than other single feature recognition methods in walking, sitting down, standing up, pushing, pulling, fault, and other actions; On this action, the recognition accuracy of the multi-feature voting human action recognition algorithm based on SOM neural network is low. On the whole, the performance of the proposed method is the best.

In Figure 8, the recognition rates of histograms of 3D joints method, skeleton joint features method, random forest fusion strip feature method, and the proposed multi-feature voting human action recognition algorithm based on SOM neural network are compared on the data set UT-Kinect action. It can be seen that the recognition rate of the skeleton joint features method is the lowest (87.90%) on the data set UT-Kinect action and the human action recognition rate of multi-feature voting based on SOM neural network is the highest (93.68%). The above results show that the construction of intelligent cultural tourism and virtual reality based on SOM neural network multi-feature voting human action recognition algorithm can identify more actions and bring more real tourism experience to users. Different from the UT-Kinect action data set, the similarity of actions on MSRDailyActivity3D data set increases, and the same actions will be collected once when standing and once when sitting, which increases the difficulty of action recognition in data set to a certain extent. In order to verify the effectiveness of the key frame action recognition scheme extracted by SOM in the study, MSRDailyActivity3D data set was selected to compare the recognition rate and time consumption of non-key frame action recognition and key frame action recognition.

As can be seen from Figure 9, the recognition rate of key frames (56.00%, 97.00%, and 93.00%) is higher than that of non-key frames (54.00%, 93.00%, and 92.00%). The key frame is extracted by SOM, and the subsequent key frame recognition is slightly lower than the non-key frame recognition. This is because data loss cannot be avoided when the key frame is extracted. However, there is little difference in the average recognition accuracy between the two, and the whole process of action recognition through key frames only takes 3.59 s, while action recognition without key frames takes 34.92 s. On the whole, key frame action recognition has more advantages. In the data set MSRDailyActivity3D, the key frame method of K-means, the fusion depth information method of joint point position, the fusion depth information of joint angle, and the proposed multi-feature voting human action recognition algorithm of SOM neural network are used to recognize each action.

As shown in Figure 10, the accuracy of motion recognition based on the K-means key frame method is 54.00%, which is higher than the accuracy of motion recognition based on joint position fusion depth information (50.00%). The accuracy of motion recognition based on joint angle fusion depth information is 57.00%, which is better than K-means key frame method. The accuracy of multi-feature voting human action recognition algorithm based on SOM neural network is 59.06%, which is the highest recognition rate among the four action recognition algorithms.

### 4.2. Analysis of Practical Application Effect of Smart Cultural Tourism Based on SOM Neural Network

A small tourism organization is selected to introduce a human-computer interactive virtual reality tourism project (represented by project a) fused with a convolutional neural network, human-computer interactive virtual reality tourism project (represented by project B) fused with joint vector naive Bayesian action recognition algorithm, human-computer interactive virtual reality tourism project (represented by project C) fused with machine learning, and human-computer interactive virtual reality tourism project (expressed as project d) with SOM neural network and other eigenvectors as the core algorithm. The four projects charge the same fees. The profitability of the Tourism Organization in the four projects and the user's evaluation score are compared.

As shown in Figure 11, when the four kinds of virtual reality tourism projects were introduced (March), there was no significant difference in the income of each project. The profit of the interactive virtual reality tourism project integrating machine learning was 61,000 yuan, slightly higher than the other three projects. In April, the profit of man-machine interactive virtual reality tourism project with convolution neural network was 4,000 yuan less than that in March, and the profit of man-machine interactive virtual reality tourism project with SOM neural network and other feature vectors as the core algorithm increased to 6,1000 yuan. Within 6 months after the introduction of the project, the human-computer interactive virtual reality tourism project integrated with convolutional neural network made a total profit of 371,000 yuan; the human-computer interactive virtual reality tourism project integrated with joint vector naive Bayesian action recognition algorithm made a total profit of 407,000 yuan; and the human-computer interactive virtual reality tourism project integrated with machine learning made a total profit of 356,000 yuan, The human-computer interactive virtual reality tourism project with SOM neural network and other eigenvectors as the core algorithm made a total profit of 422,000 yuan. To sum up, the profit of human-computer interactive virtual reality tourism project with SOM neural network as the core algorithm is higher than the other three projects.

According to the evaluation scores and contents, the user evaluation is divided into four levels. Level I refers to the dissatisfaction of users, poor experience, weak sense of reality, and the inability to give effective feedback on the actions of users in the process of use. Level II refers to that the user is relatively satisfied and can give feedback on the user's actions in the process of use, but the feedback is not timely or the feedback result does not conform to the actual operation and has a certain sense of experience. Level III refers to the user's satisfaction; the feedback can be given to the user's actions in the process of use; the feedback is timely; there are a few errors in the feedback process; and the sense of experience is good. Level IV refers to the user's satisfaction; a good sense of experience, a strong sense of reality, timely, and effective feedback for the user's actions in the process of use; and there is basically no error in the feedback.

As shown in Figure 12, the user rating of the human-computer interactive virtual reality tourism project based on convolutional neural network accounts for 26% of the total, 39% of the total, 23% of the total, and 12% of the total. The user rating of human-computer interaction virtual reality tourism project based on joint vector naive Bayes action recognition algorithm is grade I, grade II, grade III, and grade IV, accounting for 17%, 42%, 30%, and 11%, respectively. The proportion of user rating of human-computer interaction based on machine learning is 35%, 46%, 15%, and 4%, respectively. The user rating of human-computer interactive virtual reality tourism project with SOM neural network and other feature vectors as the core algorithm is 12%, 34%, 40%, and 14%, respectively. It can be seen that the human-computer interactive virtual reality tourism project with SOM neural network as the core algorithm is more popular among users, and the proportion of satisfied users and very satisfied users are higher than the other three projects. The above results show that the algorithm of multi-feature extraction based on SOM neural network can achieve rapid action recognition with high recognition accuracy, and users can get highly accurate, timely, and effective feedback in the process of using.

## 5. Conclusion

Virtual reality technology provides tourists with a real and vivid introduction of the landscape, and tourists can form a general understanding of the unfamiliar scenic spots through virtual reality technology. Although there are many effective algorithms, such as emperor butterfly optimization (MBO), earthworm optimization (EWA), elephant grazing optimization (EHO), moth search (MS) algorithm, slime mold algorithm (SMA), and Harris hawks optimization (HHO), it is undeniable that there are still few studies that combine these algorithms with virtual reality. The key technology of virtual reality tourism is human action recognition, so this paper proposes an action recognition algorithm based on SOM neural network multi-feature vector, which uses SOM neural network to obtain the key frame of tourists' action, reduces the recognition time, and combines it with multi-feature recognition method to increase the accuracy of action recognition. The results show that on the UT-Kinect action data set, the average accuracy of human action recognition algorithm based on SOM neural network multi-feature voting is 93.68%, which is higher than that of random forest fusion feature method. On the data set MSRDailyActivity3D, the time consumption of action recognition by key frame recognition is only 3.59 s, which is significantly less than that by non-key frame recognition (34.92 s). The accuracy of action recognition by multi-feature voting algorithm based on SOM neural network is 59.06%. The total profit (422,000 yuan) and user evaluation (II + III + IV) of man-machine interactive virtual reality tourism project with SOM neural network multi-eigenvector as the core algorithm are higher than those of man-machine interactive virtual reality tourism project with convolution neural network (371,000 yuan), the human-computer interactive virtual reality tourism project (407,000 yuan), and the human-computer interactive virtual reality tourism project (356,000 yuan) based on joint vector naive Bayesian action recognition algorithm and machine learning. Compared with the traditional general algorithm, the multi-feature vector recognition method based on SOM neural network proposed in this paper can achieve a better recognition effect in action recognition and bring more real experience to users. The research lacks the content of action description for the combination of multiple features, and the follow-up experiments should conduct more in-depth mining on the multi-feature features and further summarize the relationship between the target features, in order to achieve a more accurate landscape introduction.

## Figures and Tables

**Figure 1:** Flow chart of human motion feature extraction.

**Figure 2:** Skeleton structure after joint point number.

**Figure 3:** SOM neural network structure diagram.

**Figure 4:** Flow chart of key frame extraction algorithm based on SOM neural network.

**Figure 5:** Human action recognition method flow based on the voting strategy of multi-feature classification results.

**Figure 6:** SOM neural network model training results.

**Figure 7:** The recognition rate of each action under different features.

**Figure 8:** Recognition rate of different methods on UT-Kinect data set.

**Figure 9:** The recognition rate of action obtained by using non-key frame and key frame.

**Figure 10:** Recognition rate of different methods on MSRDailyActivity3D data set.

**Figure 11:** Comparison of profitability of different projects within 6 months.

**Figure 12:** Evaluation of different projects within 6 months.

## Data Availability

The data used to support the findings of this study are available from the corresponding author upon request.
